# Role of glycogen synthase kinase-3β and PPAR-γ on epithelial-to-mesenchymal transition in DSS-induced colorectal fibrosis

**DOI:** 10.1371/journal.pone.0171093

**Published:** 2017-02-16

**Authors:** Jacopo Di Gregorio, Roberta Sferra, Silvia Speca, Antonella Vetuschi, Caroline Dubuquoy, Pierre Desreumaux, Simona Pompili, Loredana Cristiano, Eugenio Gaudio, Vincenzo Flati, Giovanni Latella

**Affiliations:** 1 Department of Biotechnological and Applied Clinical Sciences, University of L'Aquila, L'Aquila, Italy; 2 University of Lille, U995, Lille Inflammation Research International Center (LIRIC), F-59000 Lille, France; 3 IBD, Lille, France; 4 CHR Lille, Service des Maladies de l’Appareil Digestif et de la Nutrition, Hôpital Claude Huriez, Lille, France; 5 Department of Life, Health and Environmental Sciences, University of L'Aquila, L’Aquila, Italy; 6 Department of Human Anatomy, University of Rome La Sapienza, Rome, Italy; 7 Department of Life, Health and Environmental Sciences, Gastroenterology Unit, University of L'Aquila, L'Aquila, Italy; National Cancer Center, JAPAN

## Abstract

**Background:**

Intestinal fibrosis is characterized by abnormal production and deposition of extracellular matrix (ECM) proteins by activated myofibroblasts. The main progenitor cells of activated myofibroblasts are the fibroblasts and the epithelial cells, the latter through the epithelial-mesenchymal transition (EMT).

**Aim:**

To evaluate the action of the new PPAR-γ modulator, GED-0507-34 Levo (GED) on the expression of EMT associated and regulatory proteins such as TGF-β, Smad3, E-cadherin, Snail, ZEB1, β-catenin, and GSK-3β, in a mouse model of DSS-induced intestinal fibrosis.

**Methods:**

Chronic colitis and fibrosis were induced by oral administration of 2.5% DSS (w/v) for 6 weeks. GW9662 (GW), a selective PPAR-γ inhibitor, was also administered by intraperitoneal injection at the dose of 1 mg/kg/day combined with GED treatment. All drugs were administered at the beginning of the second cycle of DSS (day 12). 65 mice were randomly divided into five groups (H_2_O as controls n = 10, H_2_O+GED n = 10, DSS n = 15, DSS+GED n = 15, DSS+GED+GW n = 15). The colon was excised for macroscopic examination and histological and morphometric analyses. The level of expression of molecules involved in EMT and fibrosis, like TGF-β, Smad3, E-cadherin, Snail, ZEB1, β-catenin, GSK-3β and PPAR-γ, was assessed by immunohistochemistry, immunofluorescence, western blot and Real Time PCR.

**Results:**

GED improved the DSS-induced chronic colitis and fibrosis. GED was able to reduce the expression of the main fibrosis markers (α-SMA, collagen I-III and fibronectin) as well as the pivotal pro-fibrotic molecules IL-13, TGF-β and Smad3, while it increased the anti-fibrotic PPAR-γ. All these GED effects were nullified by co-administration of GW with GED. Furthermore, GED was able to normalize the expression levels of E-cadherin and β-catenin and upregulated GSK-3β, that are all known to be involved both in EMT and fibrosis.

**Conclusions:**

The DSS-induced intestinal fibrosis was improved by the new PPAR-γ modulator GED-0507-34 Levo through the modulation of EMT mediators and pro-fibrotic molecules and through GSK-3β induction.

## Introduction

Intestinal fibrosis is one of the main complications of the Inflammatory Bowel Disease (IBD), affecting more than 30% of Crohn’s disease (CD) patients and almost 5% of Ulcerative Colitis (UC) patients [1–3]. Characterized by an uncontrolled production and deposition of extracellular matrix components (ECM), intestinal fibrosis is the main cause of lumen stricture and obstruction that can lead to loss of function of the affected digestive tracts.

To date, efficient and well-tolerated anti-fibrotic drugs are not yet available and surgery represents the only therapeutic solution for intestinal fibrosis. Indeed, the anti-inflammatory treatments, in IBD or in other chronic inflammation-associated fibrotic conditions of various organs (lung, liver, kidney) does not prevent the evolution of fibrosis once the process has started [4–7]. The lack of effective pharmacological treatments resides in the intrinsic complexity of the fibro-proliferative processes.

In order to identify potential targets for the development of efficient anti-fibrotic therapies a more accurate focus on the specific cellular mechanisms leading to the progression of fibrosis is imperative.

To date, it is well established that the ECM remodeling is one of the main activity of myofibroblasts exposed to both profibrotic and antifibrotic factors directly orchestrated by the TGF-β/Smad pathway, the major driving force of fibrosis [8].

Several evidences have demonstrated that activated myofibroblasts can derive from several and distinct cellular source, such as resident mesenchymal cells (fibroblasts, subepithelial myofibroblasts, and smooth muscle cells), as well as by stellate cells, pericytes and bone marrow stem cells [1]. In addition, activated myofibroblasts can differentiate from not-mesenchymal cells, such as epithelial or endothelial cells, via the epithelial-mesenchymal transition [EMT] or the endothelial-mesenchymal transition [EndoMT] respectively [2–3].

Several evidences have demonstrated that epithelial cells can have an impact on the development and progression of fibrosis comparable to that of the fibroblasts and, therefore, EMT may represent one of the pivotal mechanisms promoting fibro-proliferative processes.

In EMT, epithelial cells slowly gain myofibroblast markers as they lose their epithelial elements [9]. These cells then leave the epithelial layer (mainly due to the E-cadherin loss) and accumulate in the interstitium, thus beginning the ECM synthesis. At the molecular level, EMT is regulated by a complex signaling network involving the TGF-β/Smad pathway. Transcriptional activators, such as ZEB1 and Snail, seem also implied in the development of fibrosis in various organs as inhibiting factors of the E-cadherin expression [10–12]. Furthermore, the EMT process appears to be regulated by glycogen synthase kinase-3beta (GSK-3β). In fact, its inhibition causes EMT in several *in vitro* cancer models. It has been shown that GSK-3β seems to negatively regulate EMT by inhibiting the transcription factor Snail, a well-known EMT activator and E-cadherin suppressor [13]. Moreover, GSK-3β has been observed to play an anti-fibrotic effect in fibrosis models *in vitro* [14–15]. However, GSK-3β inhibition has been also associated with fibrosis reduction, in *in vivo* models of kidney and lung fibrosis [16]. Thus, GSK-3β seems to have a controversial role in fibrosis, probably depending on the pathological context. In non-fibrotic conditions, E-cadherin enters in a protein complex, with β-catenin, located at the cell-cell junctions [17]. This complex maintains epithelial cell-to-cell adhesion and its deregulation (due to E-cadherin loss and EMT) leads to a fibrotic reaction in various organs [18–21]. Thus E-cadherin downregulation may represent a valid marker of EMT.

The TGF-β/Smad pathway has been identified as one of the stronger stimuli of EMT and fibrosis. These TGF-β/Smad effects are counteracted by the peroxisome proliferator-activated receptor (PPAR)-γ [22–24]. PPAR-γ, is a member of the ligand-activated transcription factors of the nuclear hormone receptor superfamily, with pleiotropic effects on lipid metabolism, inflammation, cell proliferation and fibrosis [25].

A significantly impaired PPAR-γ expression was observed in colonic epithelial cells of IBD patients, suggesting that the disruption of PPAR-γ signaling may represent a critical step of the IBD pathogenesis [26]. Overexpression of PPAR-γ prevents tissue fibrosis, whereas its loss increases fibrosis [8]. Furthermore, PPAR-γ agonists attenuate fibrosis in several organs including the intestine and these anti-fibrotic effects are abolished by PPAR-γ selective antagonists [8, 24, 25, 26]. On these basis PPAR-γ appears to be an innate protector against excessive fibrogenesis.

Recently, it has been reported that a new PPAR-γ modulator, GED-0507-34 Levo (GED), ameliorated intestinal fibrosis in dextran sulfate sodium-induced chronic colitis in mice (DSS mice) and inhibited *“in vitro”* the TGF-β–induced differentiation, both of intestinal fibroblast and epithelial cells into activated ECM-producing myofibroblasts [24].

We hypothesized that the TGF-β/Smad3 pathway, E-cadherin, β-catenin, ZEB1, Snail, GSK-3β and PPAR-γ may act as a complex signaling network, with extensive crosstalk and strong effects on EMT and intestinal fibrosis.

Therefore, in this study, we evaluated *“in vivo”* the activity of the new PPAR-γ modulator, GED-0507-34 Levo (GED), on all these EMT-associated mediators, in a mouse model of DSS-induced intestinal fibrosis.

## Materials and methods

The study has been performed at the Institution of Pasteur Animal care facility (Institut Pasteur de Lille, France) according to governmental guidelines and approved by the “Comité d’Ethique en Expérimentation Animale Nord-Pas de Calais” (CEEA n°75; ethic committee for animal experimentation of the region Nord-Pas de Calais–France).

### Animals

A total of 65 wild-type C57BL/6 mice, purchased from Janvier (Le Genest-St-Isle, France), were included in the study. All mice were maintained in a specific pathogen-free facility, fed with a standard diet and given free access to water under constant room temperature with a 12h light/12h dark cycles. Animal experiments were performed according to the governmental guidelines N° 68/609/CEE. The mice were generally euthanized three days after the third cycle of DSS when the colitis was fully induced. DSS-induced chronic colitis in mice could cause 20% of death due to the loss of weight and diarrhea. In order to prevent unnecessary suffering for the animals, the mice were euthanized earlier and in particular when their weight loss was more than 20% of their initial weight. The mice were anesthetized by isoflurane only at the time of euthanasia.

### Induction and evaluation of chronic colitis

Chronic colitis and fibrosis were induced in mice by oral administration of 2.5% (w/v) DSS (MW: 36,000–44,000, purchased from TdB Consultancy, Uppsala, Sweden) resuspended in autoclaved tap water and administered *ad libitum* for three cycles (5 days DSS followed by 7 days of tap water). Control groups received tap water only. Animals were monitored daily for fluid intake, weight changes, and examined for signs of colitis including weight loss, diarrhea (scored on a 0–2 scale, as follows: 0 = absence, 1 = mild, 2 = severe), rectal bleeding, assessed with the ColoScreen III Lab Pack (Elitech, Salon-de-Provence, France) and prolapse, (scored as 0 = absence, 1 = presence).

### Experimental design

The mice were randomly divided into five groups. Group A: control (H_2_O) n = 10, group B: H_2_O+GED n = 10, group C: DSS n = 15, group D: DSS + GED n = 15, group E: DSS+GED+GW n = 15. GED-0507-34 Levo (purchased from Nogra Pharma Ltd, Dublin, Ireland) was dissolved in a solution containing 0.5% carboxymethylcellulose sodium salt (CMC; MW 90,000 Da; Sigma-Aldrich, Milano, Italy) and 1% Tween 80 and administered at the dose of 30mg/Kg/day by oral gavage (100μl/mouse). This dose was chosen based on the results of a preliminary study carried out to identify the best dose-response effect and safety of the drug. GW9662 (GW) (Sigma-Aldrich), a selective PPAR-γ inhibitor, was also administered, combined with GED, by intraperitoneal injection at the dose of 1 mg/kg/day. All drugs were administered at the beginning of the second cycle of DSS (day 12). The control groups were orally administered with daily equal volume of vehicle.

### Samples recovery and preparation

Four days after the last DSS cycle administration, the animals of each group were euthanized by cervical dislocation under deep CO_2_ anaesthesia and underwent to laparotomy. The colon and rectum were visualized and rapidly excised. The presence of adhesions between the colon-rectum and adjacent organs was scored on a 0–2 scale [27]. The length and weight of the colon and rectum were measured and then scored for macroscopic lesions. The colonic tissue samples were subsequently fixed in 4% buffered formaldehyde and embedded in paraffin for histological and immunohistochemistry analyses. The remaining tissue specimens were stored at −80°C for Western blot and Real Time PCR analysis.

### Assessment of macroscopic and microscopic colonic lesions

The colonic length and weight were measured and then scored for macroscopic lesions. The macroscopic colonic lesions were scored by two independent observers (S.S. and C.D.) who were unaware of the treatment. They assessed and scored the individual macroscopic colonic lesions on a 0–2 scale, as follows: colonic adhesions (0 = absence, 1 = mild/focal zonal, 2 = severe/diffuse); colonic dilation (0 = absence, 1 = mild, 2 = severe); colonic thickness (0 = normal, 1 = mild increase, 2 = marked increase, > 3 mm) [27]. The sum of the scores of colonic lesions was expressed as total macroscopic score. Interobserver agreement was 95% for all appointed score.

Colonic specimens of all animals were washed and immediately fixed in 4% buffered formalin in phosphate buffer saline (PBS) at pH 7.4 for 3h at room temperature followed by the standard procedure for paraffin embedding. Serial 3-μm sections were stained with Haematoxylin and Eosin (H&E), to assess the degree of inflammation, and with Masson’s Trichrome, to detect connective tissue and fibrosis. The stained sections were then observed under an Olympus BX51 Light Microscope (Olympus Optical Co. Ltd, Tokyo, Japan). Two pathologists (A.V. and R.S.) independently examined and scored all histological sections of the colonic samples in double-blind, according to the presence of ulcerations (0 = absent, 1 = small ulcers, 2 = big ulcers), degree of inflammation (0 = absent, 1 = mild, 2 = moderate and 3 = severe), depth of the lesions (0 = absent, 1 = lesions extending in the submucosa, 2 = lesions in the muscolaris propria and 3 = lesions in the serosa) and degree of fibrosis (0 = absent; 1 = mild, 2 = moderate and 3 = severe). The sum of these scores was expressed as total microscopic score as previously reported [27]. The degree of intestinal inflammation was scored as absent, mild, moderate or severe, according to the density and extent both of the acute and chronic inflammatory infiltrate, loss of goblet cells, and bowel wall thickening. Intestinal fibrosis was scored as mild, moderate or severe, depending on the density and extent of trichrome-positive connective tissue staining and disruption of tissue architecture, as previously described [27]. Quantitative comparison of Masson’s stainings were measured by the ImageJ digital image analysis public domain software (W. S., Rasband, Image J, U. S. National Institutes of Health, Bethesda, MD; http://rsb.info.nih.gov/ij/, 1997–2011). The staining was expressed as a percentage of the total software-classified areas and the data obtained were plotted as histograms.

### Immunohistochemistry and immunofluorescence

Tissue specimens from the colon were dissected and fixed in 4% buffered formalin, in phosphate buffer saline (PBS, pH 7.4) solution for 3 hours at room temperature; they were dehydrated in a graded ethanol series, and embedded in low-temperature-fusion paraffin. 3-μm-thick sections were incubated in methanol for 40 min and then in 3% hydrogen peroxide for 5 min.

Samples were left to incubate overnight at 4°C with specific antibodies against PPAR-γ (sc-7273), TGF-β (sc-146), Smad3 (sc-6202), α-SMA (sc-32251), Collagen I-III (sc-8784; 8781), β-catenin (sc-7199) and E-cadherin (sc-7870) (Santa Cruz Biotechnology Inc., Santa Cruz, CA, USA), used at dilution of 1:200, 1:400, 1:200, 1:200, 1:400, 1:100 and 1:100 respectively, in PBS. Fibronectin (A0245, Dako Italia, Milano, Italy), was used at dilution of 1:200 (CTRL and DSS+ GED) and 1:100 (DSS), in PBS. The samples were washed for 5 min with PBS and incubated with streptavidin-biotin-peroxidase conjugated secondary antibody (K0675, Dako-Cytomation, Milano, Italy). After one wash in PBS for 10 min the sections were subject to incubation with 3,3-diaminobenzidine-tetrahydrochloride for 1–3 min. The specificity of the immune reaction was revealed by omitting the primary antibodies. Finally the samples were stained with Hematoxylin of Mayer and observed under the Olympus BX51 Light Microscope (Olympus, Optical Co. Ltd., Tokyo, Japan).

For immunofluorescence (IF) staining, non-specific protein binding was blocked with 10% Bovine Serum Albumin (BSA) in PBS for 2 hours at room temperature. Sections were incubated overnight at 4°C with mouse anti β-catenin (sc-7963) and rabbit anti E-cadherin (sc-7870) (Santa Cruz Biotechnology Inc., Santa Cruz, CA, USA) used at dilutions of 1:300. After rinsing in PBS for 10 minutes for three times, section were incubated with goat anti-rabbit Alexa Fluor 633 for E-caderin and goat anti-mouse Alexa Fluor 488 for β-catenin (Thermo Fisher Scientific Inc). All secondary antibodies were diluted (1:2000) and incubated at room temperature for 2 hours. Negative controls (the primary antibody was replaced with preimmune serum) were included for all immunoreactions. Sections were treated with mounting medium from Vector Laboratories containing DAPI and photographed through a Leica TCS SP2 (Leica, Manheim, Germany) confocal microscope.

### Quantitative digital image analysis of immunohistochemical staining

Quantitative comparison of immunohistochemical stainings were measured by the ImageJ digital image analysis public domain software (W. S., Rasband, Image J, U. S. National Institutes of Health, Bethesda, MD; http://rsb.info.nih.gov/ij/, 1997–2011). The IHC profiler software plugin was required. The immunopositivity was expressed as a percentage of the total software-classified areas and the data obtained were plotted as histograms.

### Western blot

Total proteins were extracted from colon tissues in lysis buffer (50 mM Tris.Cl pH 7.8, 1% Triton X100, 0.1% SDS, 250 mM NaCl, 5 mM EDTA, 100 mM NaF, 2 mM NaPPi, 2 mM Na3VO4, 1 mM PMSF, 1mM Aprotinin, 1mM Pepstatin, 1mM Leupeptin). The crude lysate was centrifuged at 16000 g for 15 minutes, the supernatant was recovered and assayed for protein concentration by the Bradford Assay (Bio-Rad Laboratories, Milano, Italy). The nuclear protein extracts were obtained from the colon tissues by using the NXTRACT kit (Sigma-Aldrich, Milano, Italy), according to the manufacturer’s instructions.

The protein extracts were run on a 10% SDS-PAGE for β-catenin, E-cadherin, (phosphor-Y216) GSK-3β, GSK-3β, Snail and ZEB1 analyses and transferred onto a PVDF membrane (Millipore, Milano, Italy). The membranes were stained with Ponceau Red (Sigma-Aldrich, Milano, Italy), in order to verify the proper protein transfer, and were blocked at RT for 1 hour with 5% non-fat dry-milk in TBST containing 0.1% Tween20. After this, the membranes were washed briefly and incubated with primary antibodies (purchased from Santa Cruz Biotechnology, Heidelberg, Germany, and Abcam, Cambridge, UK) directed either against β-catenin (1:1000, O/N at 4°C), E-cadherin (1:1000 O/N at 4°C), ZEB1 (1:1000, O/N at 4°C), Snail (1:1000, O/N at 4°C), p-GSK-3β (1:1000, O/N at 4°C) and GSK-3β (1:1000, O/N at 4°C) diluted in 5% non-fat milk in TBST 0.1% Tween20.

The membranes were then washed three times for 10 minutes with TBST. Then, they were incubated for 1 hour at room temperature (RT), with anti-rabbit or anti-mouse (depending on the primary antibody) HRP-conjugated secondary antibody (Bio-Rad Laboratories, Milano, Italy) diluted 1/2000 in TBST containing 5% non-fat milk. The membranes were washed 3 times for 10 minutes, incubated in SuperSignal West Pico (Thermo Fisher Scientific Inc, Rockford, IL, USA) chemiluminescent substrate and detected using a ChemiDoc XRS-plus imaging system (Bio-Rad Laboratories, Milano, Italy). The optical densities of the blot bands were finally determined using a computer-assisted densitometer (ImageJ, U. S. National Institutes of Health, Bethesda, Maryland, USA) and normalized versus the β-actin (sc-1616) or vinculin (sc-5573) internal controls (Santa Cruz Biotechnology, Heidelberg, Germany).

### Real time PCR

RNA was extracted from colon tissues using the NucleoSpin RNA kit (Macherey-Nagel, Hoerdt, France), then 1 μg of RNA was retro-transcribed into cDNA using a High Capacity cDNA Reverse Transcription Kit (Applied Biosystems, Foster City, CA, USA) according to the manufacturer's protocol, and the equivalent of 0.1 μg was used for the quantitative real-time PCR reactions by using the Power SYBR® Green PCR Master Mix (Applied Biosystems, Foster City, CA, USA) on a StepOne Real-Time PCR System (Applied Biosystems, Foster City, CA, USA). Primers sets included Acta2 for α-SMA, Fn1 for Fibronectin, COL1a1 for Collagen I-III, Il-13 for IL-13, Tgfb 1 for TGF-β1, Smad3 for SMAD3 and Pparg for PPAR-γ. A critical threshold cycle (Ct) value, was determined for each reaction. Relative gene expression values were calculated as E = 2^-ΔCt^, where ΔCt is the difference in crossing points between the housekeeping gene, GAPDH, and each target gene. The primers for each gene are listed in Table 1.

**Table 1:** Primer sequences used for quantitative RT-PCR analysis.

Gene	Source	Primer	Sequences (5’ → 3’)
Acta2	Mouse	Forward	CCT GAC GGG CAG GTG ATC
		Reverse	ATG AAA GAT GGC TGG AAG AGA GTC T
COL1a1	Mouse	Forward	GAG TAC TGG ATC GAC CCT AAC CAA
		Reverse	ACA CAG GTC TGA CCT GTC TCC AT
Fn1	Mouse	Forward	CGAAGCCGGGAAGAGCAAG
		Reverse	CGTTCCCACTGCTGATTTATCTG
GAPDH	Mouse	Forward	ATG GGA AGC TTG TCA TCA ACG
		Reverse	GGC AGT GAT GGC ATG GAC TG
IL-13	Mouse	Forward	CAG TCC TGG CTC TTG CTT G
		Reverse	CCA GGT CCA CAC TCC ATA CC
TGF-β1	Mouse	Forward	CCC GAA GCG GAC TAC TAT GCT
		Reverse	GTT TTC TCA TAG ATG GCG TTG TTG
Smad3	Mouse	Forward	TGG ACT TAG GAG ACG GCA GTC C
		Reverse	CTT CTG AGA CCC TCC TGA GTA GG
PPAR-γ	Mouse	Forward	TTG CTG AAC GTG AAG CCC ATC GAG G
		Reverse	GTC CTT GTA GAT CTC CTG GAG CAG

### Statistical analysis

Statistical analyses were performed using Kruskal-Wallis non parametric ANOVA. Post-hoc comparisons between pairs of groups were assessed by using Wilcoxon rank sum test. Results were expressed as means ± SEM. A p-value < 0.05 was considered statistically significant.

## Results

### DSS-induced chronic colitis and fibrosis are improved by PPAR-γ agonist

#### Clinical findings and macroscopic features of DSS-induced chronic colitis

DSS administration was associated with a moderate body-weight loss. Mortality was observed in 13% of mice receiving DSS and in none of the DSS mice treated with GED (Table 2).

**Table 2:** Effects of oral GED treatment on macroscopic features of DSS-induced chronic colitis in mice.

Parameters	H_2_O	H_2_O+GED	DSS	DSS+GED		DSS+GED+GW
**Duration of DSS administration (days)**	0	0	36		36	36
**Duration of GED and GW treatment (days)**	0	24	0		24	24
**Number of mice**	10	10	15		15	15
**Mortality (n.mice)**	0	0	2		0	0
**Body weight**	28,95 ± 0,331	25,73 ± 1,284	25,41 ± 0,154**		25,12 ± 0,245**	22,29 ± 1,115***
**Colon weight**	0,171 ± 0,005	0,154 ± 0,0074	0,281 ± 0,002**		0,269 ± 0,004**	0,2545 ± 0,014**
**Colon length**	0,99 ± 0,015	0,98 ± 0,04	0,786 ± 0,013**		0,828 ± 0,0085**/^¥¥^	0,709 ± 0,022**
**Colon weight/size ratio**	1,012 ± 0,02	0,9684 ± 0,042	2,151 ± 0,054**		1,661 ± 0,085*/^¥^	2,061 ± 0,14*
**Dilatation**	np	np	1,21 ± 0,13**		1,02 ± 0,15*/^¥¥^	1,3 ± 0,26**
**Thickness**	np	np	1,24 ± 0,132**		0,68 ± 0,108**/^¥^	1,7 ± 0,21**
**Stenosis**		np	0,842 ± 0,121**		0,51 ± 0,114**	0,985 ± 0,27**
**Adhesions**	np	np	0,87 ± 0,18**		0,41 ± 0,11^¥^	1,5 ± 0,26**
**Total macroscopic score**	np	np	3,106 ± 0,254		2,19 ± 0,258**/^¥¥^	4,5 ± 0,58***

Data are expressed as mean ± SEM

np = not present

* = p< 0.05 vs H_2_O

** = p< 0.01 vs H_2_O

*** = p< 0,005 vs H_2_O

^¥^ = p< 0.05 vs DSS

^¥¥^ = p< 0,01 vs DSS

DSS mice showed a significant increase of colon weight (referred to the last 8 cm of the distal large bowel) and a reduction of colon length compared to the control group. The ratio weight/length of the colon, a further indicator of inflammation and fibrosis, was markedly increased in the DSS-receiving mice compared to the control mice and it was improved by GED treatment. The main macroscopic features related to the DSS-induced fibrosis, including dilation, thickness, stenosis and adhesion, were also all improved by GED oral administration. Total macroscopic score was lower in GED-treated DSS mice compared to untreated DSS mice (2.190 ± 0.258 vs 3.106 ± 0.254, respectively, p< 0.01) (Table 2). DSS mice simultaneously treated by GED and GW, did not show improvement of colonic parameters and lesions associated to the chronic DSS administration, neither a decrease of the total macroscopic score compared to DSS group.

### Microscopic features of DSS-induced chronic colitis

Colorectal specimens from mice receiving DSS showed diffuse signs of both inflammation and fibrosis that were assessed by H&E and Masson’s Trichrome stainings, respectively (Fig 1). Inflammation involved mucosal and submucosal layers and was characterized by increased infiltrate of inflammatory cells, decrease of goblet cells, reduction and alteration of crypt architecture and presence of erosions and ulcerations. An increase of collagen deposition in the mucosa, submucosa and serosa was also observed. GED administration ameliorated the microscopic signs of both colorectal inflammation and fibrosis in DSS treated mice, but not in DSS+GED+GW treated mice (Fig 1).

**Fig 1:** Degree of colonic inflammation and fibrosis, assessed by H&E and Masson Trichrome stainings. DSS and DSS+GED+GW treated mice showed signs of severe chronic inflammation and marked fibrosis when compared to H_2_O, H_2_O+GED and DSS+GED treated mice. Original Magnification: 10X. Scale bars: 100μ.

#### α-SMA, collagen I-III, fibronectin, IL-13, TGF-β, and Smad3 are increased while PPAR-γ is decreased in DSS-induced intestinal fibrosis

The main fibrotic markers, α-SMA, collagen I-III and fibronectin, and also the pivotal pro-fibrotic molecules IL-13, TGF-β, and Smad3 and the anti-fibrotic PPAR-γ were assessed by immunohistochemical and RT-PCR assays.

Quantitative evaluation of immunohistochemical staining showed a significantly increased expression of α-SMA, collagen I-III and fibronectin in mice with DSS-induced chronic colitis and DSS+GED+GW compared to H2O controls and H_2_O + GED mice (Fig 2). α-SMA was not only localized in the typical tissue layers, such as muscolaris mucosae and muscolaris propria, but also in the lamina propria, submucosa and serosa (Fig 2). In mice receiving DSS and DSS+GED+GW a parallel increase of α-SMA, collagen I-III and fibronectin mRNA was found (Fig 3). Daily oral GED administration, in mice with DSS-induced chronic colitis, reduced all these markers of fibrosis, both at protein and mRNA level (Figs 2 and 3). DSS administration also led to a significant increase in the expression of IL-13, TGF-β1 and Smad3; this increased expression, instead, was not observed in mice with DSS-induced chronic colitis treated with GED (Figs 4 and 5). Both the immunohistochemical (Fig 6A and 6B) and the RT PCR analysis (Fig 6C) showed that PPAR-γ was less expressed in mice receiving DSS and DSS+GED+GW compared to control mice. On the other hand, the expression of PPAR-γ was significantly increased in mice with DSS-induced chronic colitis treated with a daily oral GED administration. The expression of PPAR-γ was also significantly increased in H_2_O + GED mice, especially at the mRNA level.

**Fig 2:** Immunohistochemical analysis of α-SMA, collagen I-III and fibronectin. The microphotograph (**A**) and the quantitative analysis (**B**) showed a significant reduction of α-SMA, collagen I-III and fibronectin expression in the DSS mice treated with GED compared to DSS and DSS+GED+GW mice. In DSS+GED mice the immunostaining pattern was similar to H2O controls and H_2_ O+ GED. Original Magnification: 10X. Scale bars: 100μm.

**Fig 3:** Real Time PCR analysis of the mRNA for α-SMA, collagen I-III and fibronectin. GED improved the mRNA expression of the main markers of fibrosis in DSS-induced chronic colitis in mice. Data are presented as mean of fold changes vs CTRL.

**Fig 4:** Immunohistochemical analysis of IL-13, TGF-β and Smad3. The microphotograph (**A**) and the quantitative analysis (**B**) showed an upregulation of all three examined markers in colonic wall of DSS and DSS+GED+GW treated mice compared to H_2_O controls, H_2_O+ GED and DSS + GED groups. Original Magnification: 10X Scale bars: 100μm.

**Fig 5:** Real Time PCR analysis of the mRNA for IL-13, TGF-β and Smad3. GED reduced the mRNA levels for IL-13, TGF-β, Smad3 in DSS-induced chronic colitis in mice. Data are presented as mean of fold changes vs CTRL.

**Fig 6:** Immunohistochemical and Real Time PCR analysis of PPAR-γ. The microphotograph (**A**), the quantitative analysis (**B**) and the Real Time PCR analysis (**C**) showed that in DSS and DSS+GED+GW treated mice the expression of PPAR-γ was very low, whereas in DSS+GED treated mice the expression of PPAR-γ was restored and it was similar to the levels observed in H_2_O normal control. Original Magnification: 10X. Scale bars: 100μm. Data are presented as mean of fold changes vs CTRL.

#### E-cadherin, ZEB1, Snail, β-catenin, and GSK-3β expression is modulated by a PPAR-γ agonist

E-cadherin forms a complex with β-catenin thus contributing to maintain the epithelial stability. This complex appears to be dysregulated in fibrosis. Thus, E-cadherin and β-catenin may be used as EMT markers in intestinal fibrosis and potentially as markers of disease progression as well. Instead, GSK-3β appears to act as an EMT inhibitor in the intestine.

Immunohistochemistry analysis showed that E-cadherin and β-catenin expression was predominant in the mucosa especially in the cytoplasm of the epithelial cells (Figs 7 and 8). Immunostaining for both proteins was lower in DSS and DSS+GED+GW treated mice compared to H_2_O controls and to H_2_O+GED and DSS+GED. Daily oral GED administration was able to normalize the expression levels of the two proteins. A higher level of E-cadherin and β-catenin in control mice was also confirmed by immunofluorescence analysis, in fact, while it was low in DSS mice, it increased after treatment with GED. Furthermore, in DSS mice, β-catenin appeared to be, at least in part, localized in the nucleus. (Figs 9 and 10).

**Fig 7:** E-cadherin expression is reduced in intestinal fibrosis and restored by a PPAR-γ agonist. Immunohistochemical analyses of E-cadherin (Original magnification: 40X). E-cadherin protein expression increased in H_2_O+GED and DSS+GED groups showing a similar pattern to the H_2_O controls. E-cadherin immunostaining was lower in DSS and DSS+GED+GW mice. Scale bars: 25 μm.

**Fig 8:** β-catenin is down-regulated in intestinal fibrosis. Immunohistochemical analyses of β-catenin (Original magnification: 40X). β-catenin protein expression was upregulated by GED administration in DSS and in H_2_O+GED treated mice, finding not observed in DSS and DSS+GED+GW mice. Scale bars: 25 μm.

**Fig 9:** Immunohistochemical analysis of β-catenin. β-catenin appeared to be, at least in part, localized in the nucleus in DSS mice (Original magnification: 40X). Scale bars: 25 μm.

**Fig 10:** Confocal analyses of E-cadherin and β-catenin. The immunostaining of the protein complex was significantly increased in DSS+GED group compared to the controls. In DSS group the expression was lower and β-catenin appeared to be, at least in part, localized in the nucleus, mainly, of epithelial cells.

These results were in accordance with those obtained by western blot analysis (Figs 11 and 12).

**Fig 11:** E-Cadherin Protein levels are reduced in DSS-induced chronic colitis in mice and restored by a PPAR-γ agonist. (**A**) Western Blot analysis of total E-cadherin protein levels on the five mice groups (H_2_O, H_2_O +GED, DSS+GED+GW, DSS, DSS+ GED). The lower band, indicated by an arrow, corresponding to the mature form of E-cadherin, was used for the densitometric analysis, with β-actin as internal control. (**B**) Densitometric analysis of mature E-cadherin protein levels on the five mice groups (H_2_O, H_2_O+GED, DSS+GED+GW, DSS, DSS+ GED). A significant down-regulation (p = 0,019) of E-cadherin was observed in the DSS and DSS+GED+GW groups compared to H_2_O and H_2_0+GED controls. GED administration restored E-cadherin levels (p = 0.03) compared to DSS. Data are presented as mean of fold changes vs CTRL.

**Fig 12:** β-catenin modulation in DSS-induced chronic colitis in mice. (**A**) Western blot analysis of the β-catenin protein levels on three of the five mice groups (H_2_O, DSS, DSS+GED). β-actin was used as internal loading control. (**B**) Densitometric analysis of the β-catenin protein levels on the three mice groups (H_2_O, DSS, DSS+GED). A β-catenin down-regulation was observed in the DSS group. GED administration restored the β-catenin protein levels (p = 0.026) when compared to the DSS mice. Data are presented as mean of fold changes vs H_2_O controls. (**C**) Western Blot analysis of β-catenin nuclear protein levels on the five mice groups (H_2_O, DSS, DSS+GED, H_2_O+GED, DSS+GED+GW), with β-actin as internal control. (**D**) Densitometric analysis of β-catenin nuclear protein levels. A significant β-catenin up-regulation was observed in the DSS-treated mice when compared to the H_2_O controls (p = 0,03) and to DSS+GED mice (p = 0,01). Data are presented as mean of fold changes vs CTRL.

The E-cadherin protein level was evaluated by western blot analysis on the five mice groups. We observed a significant decrease of mature E-cadherin in mice receiving DSS and DSS+GED+GW, compared to H_2_O controls and H_2_O+GED (Fig 11). GED treatment caused a restoration of E-cadherin, thus exerting a reversion of the fibrotic phenotype to the normal phenotype. In addition, GW successfully inhibited GED activity, showing that GED activity is mediated by PPAR-γ.

In order to verify if the decreased E-cadherin protein expression in DSS mice was the consequence of a regulation at the transcription level, we evaluated the E-cadherin mRNA on three (H_2_O, DSS and DSS+GED) of the five groups of mice through RT-PCR (Fig 13). The E-cadherin transcript was only slightly reduced in DSS mice, the variation between the mice groups, was not significantly different, thus it was considered not sufficient to support a transcriptional mechanism of regulation of E-cadherin expression.

**Fig 13:** Transcriptional regulation of E-cadherin in DSS-induced chronic colitis in mice. (**A**) Real-Time PCR analysis of E-cadherin mRNA levels on the three (H_2_O, DSS, DSS+ GED) of the five mice groups. The E-cadherin mRNA level was reduced, but not significantly, by DSS, compared to H_2_0 and DSS+GED. (**B**) Western Blot analysis of ZEB1 and Snail nuclear protein levels on the five mice groups (H_2_O, DSS, DSS+GED, H_2_O+GED, DSS+GED+GW), with β-actin as internal control. (**C**) Densitometric analysis of ZEB1 nuclear protein levels. A significant (p = 0,035) ZEB1 down-regulation was observed in the DSS+GED-treated mice compared to the DSS (p = 0,039) and DSS+GED+GW mice. Data are presented as mean of fold changes vs CTRL. (**D**) Densitometric analysis of Snail nuclear protein levels. A significant Snail up-regulation was observed in the DSS-treated mice compared to the H_2_O controls (p = 0,035) and to DSS+GED (p = 0,032). Similar high levels of Snail were observed in DSS+GED+GW mice. Data are presented as mean of fold changes vs CTRL.

To strengthen this result, we evaluated the nuclear protein levels of ZEB1 and Snail, the E-cadherin transcriptional regulators, both able to inhibit its expression, and associated with EMT initiation and fibrosis in other organs.

Nuclear Snail and ZEB1 protein level was evaluated by western blot analysis on the five mice groups. We saw a significant Snail induction in DSS-treated mice compared to the control groups, a finding that was significantly reversed by the GED treatment. For ZEB1 we saw a similar trend, with a significant ZEB1 reduction in DSS+GED mice compared to DSS mice (Fig 13). Paired with the E-cadherin down-regulation at the protein level, these data suggest an EMT induction in our mouse model of intestinal fibrosis, where the process is reversed by the GED treatment. This was utterly proven by the GED inhibition, obtained by using GW, where the levels of EMT markers were similar to those observed in the DSS treated mice.

The β-catenin protein level was evaluated by western blot analysis on H_2_O, DSS and DSS+GED mice groups. We found a significant β-catenin down-regulation in DSS mice and a restoration of β-catenin levels in the DSS mice treated with GED (Fig 12). The β-catenin protein levels appeared to follow the same trend of E-cadherin protein levels, suggesting an EMT-mediated disruption of the E-cadherin/β-catenin complex in fibrosis.

Furthermore, western blot analysis showed an increase of β-catenin at nuclear levels in the DSS-treated mice, thus suggesting a β-catenin nuclear translocation (Fig 12) associated with fibrosis. This event could be related to an inactive GSK-3β. In fact, when GSK-3β is not activated, β-catenin is not phosphorylated and thus it is not degraded by the proteasome in the cytoplasm, as observed in the fibrotic condition, allowing its translocation in the nucleus where it can regulate the transcription of fibrosis related genes.

On this basis the protein levels of GSK-3β and the levels of its active, phosphorylated at Tyr216, form were evaluated by western blot analysis in the H_2_O, DSS and DSS+GED groups. GSK-3β phosphorylation at Tyr216 was significantly increased in DSS mice treated with GED, compared to both the control and the untreated DSS mice (Fig 14). Thus, it can be inferred that GSK-3β activation may be required for the restoration of the epithelial phenotype exerted by GED treatment in the intestine, possibly by promoting the stability of the E-cadherin/β-catenin complex. Preliminary results showed an increase of GSK-3β phosphorylation at Tyr216 also in the control mice treated with GED, showing that such action of the GED is, at least in part, independent from DSS (data not shown).

**Fig 14:** GED markedly increased the GSK-3β phosphorylation in DSS-induced chronic colitis in mice. (**A**) Western blot analysis of phospho-GSK-3β and GSK-3β protein levels on three of the five mice groups (H_2_O, DSS, DSS+GED). Vinculin was used as internal loading control. (B) Densitometric analysis of GSK-3β phosphorylation (phospho-GSK-3β/GSK-3β ratio). A strong (p = 0.0006) GSK-3β phosphorylation was observed in the GED group compared to the H_2_0 and DSS groups, whereas there were not significant modulations between the latter two groups. Data are presented as mean of fold changes vs CTRL.

## Discussion

In contrast to the intensive investigations focusing on the immunological mechanisms related to the early phases of intestinal inflammation and repair, the pathophysiology of chronic mucosal wound healing and the late events of repair leading to intestinal fibrosis remain largely unexplored [8, 28, 29]. Consequently, this lack of knowledge has contributed to the lack of development of effective anti-fibrotic drugs and the fact that the intestinal fibrosis still is a frequent indication for surgery in several enteropathies, especially in Crohn’s disease.

Intestinal fibrosis is characterized by abnormal production and deposition of ECM proteins by activated myofibroblasts, which are modulated by both profibrotic and antifibrotic factors [29]. Whereas in other organs the source of ECM- producing myofibroblasts is restricted to a few cell types, in gastrointestinal system the situation is more complicated as multiple cell types may become activated ECM-producing myofibroblasts [2–3]. In liver fibrosis, besides hepatic stellate cells and hepatocytes, during experimental biliary injuries (BDL) cholangiocytes are also involved in EMT process. Impairment of neuropeptide, gastrointestinal hormones and growth factors leads to cholangiocites growth/loss alterations and changing in cell morphology and function that could be partially ameliorate pharmacologically [30,31].

In intestinal fibrosis, the main progenitor cells of activated myofibroblasts are the fibroblasts and the epithelial cells, the latter through the process of EMT [2,3,12].

Myofibroblasts are activated by a variety of mechanisms including paracrine signals derived from immune and nonimmune cells, autocrine factors secreted by myofibroblasts, pathogen-associated molecular patterns derived from microorganisms that interact with pattern recognition receptors such as Toll-like receptors, and the so called damage-associated molecular patterns (DAMPs) derived from injured cells [8, 29]. Fibrosis also depends on the balance between the production and degradation of ECM proteins [29,32,33]. All these factors are directly orchestrated by the TGF-β/Smad pathway, that is considered the”core pathway” of fibrosis, and several evidences have demonstrated its strong involvement in the cellular changes due to EMT [8]. Nevertheless, several profibrogenic and antifibrogenic molecules seem to interact directly with the TGF-β/Smad pathway. The specific interaction between TGF-β/Smad3 pathway and other molecules involved in EMT and fibrosis, like E-cadherin, ZEB1, Snail, β-catenin, GSK-3β, and PPAR-γ, is still unclear.

In our model of DSS-induced chronic colitis and fibrosis in mice, we showed a marked increase in α-SMA (a marker of activated myofibroblasts), collagen I-III, and fibronectin and a parallel increased expression of pro-fibrotic IL-13, TGF-β and Smad3, compared to control mice. On the other hand, PPAR-γ, E-cadherin and β-catenin were reduced in the same DSS mice. The ZEB1 nuclear protein level was induced by DSS, but not significantly. Instead the nuclear level of the transcription factor Snail was significantly induced in DSS treated mice. The total GSK-3β protein level was not significantly changed. The new PPAR-γ modulator GED-0507-34 Levo improved the DSS-induced intestinal fibrosis through the modulation of EMT markers and pro-fibrotic molecules. Daily oral administration of GED significantly reduced the main markers of fibrosis, represented by α-SMA, collagen I-III, and fibronectin, as well as the pro-fibrotic IL-13, TGF-β and Smad3, increased PPAR-γ, restored the EMT markers, such as E-cadherin and β-catenin, significantly reduced the levels of nuclear Snail and ZEB1, and strongly activated GSK-3β. These effects, induced by GED treatment, were reverted by the concomitant administration of the irreversible PPAR-γ inhibitor GW.

The mechanisms by which the enhanced PPAR-γ signaling inhibit EMT and fibrosis are not yet fully defined. Activation of PPAR-γ by either naturally occurring or synthetic ligands can inhibit the induction of profibrotic responses induced by TGF-β, including the EMT process [34]. Agonistic activation of PPAR-γ may attenuate TGF-β1 induced EMT by acting both on Smad and non-Smad signaling TGF-β pathways. Smad2 and Smad3 phosphorylation is important for initiation of TGF-β signaling associated with EMT process, but this finding was not evaluated in this study. In hepatic stellate cells, PPAR-γ ligands prevented Smad3 phosphorylation [35]. In contrast, in the TGF-β-mediated fibroblast activation, PPAR-γ agonists did not prevent Smad2/3 phosphorylation or nuclear accumulation, but, instead, prevented recruitment of the coactivator p300 to the transcriptional complex [36]. PPAR-γ ligands also ameliorates EMT and fibrosis through the modulation of several other pathways including the tumor suppressor phosphatase and tensin homolog (PTEN), mitogen-activated protein kinases (p38, ERK1/2), early growth response-1 (Egr1), PI3K/Akt, Wnt/β-catenin, E-cadherin, Snail, ZEB1, and GSK-3β, as well as through specific miRNA [8,29,34, 37, 38, 39, 40].

The E-cadherin downregulation in the fibrotic mice, that we have observed, is consistent with the EMT process as the main source of myofibroblasts in intestinal fibrosis.

We have also observed that EMT progresses with the disease and restoration of the epithelial phenotype via GED treatment, also restores E-cadherin levels. Both E-cadherin induction and its inhibition (reflected by EMT and the consequent fibrosis) seem to be modulated at the transcription level, according to the Snail and ZEB1expression levels in the nuclei, although our Real-Time PCR assay does not show a statistically significant modulation of E-cadherin mRNA in the three mice groups.

The epithelial stability is generally maintained by the complex that E-cadherin forms with β-catenin [17]. In our study, we show a similar trend for E-cadherin and β-catenin protein expression, both immunohistochemical and western blot analysis, underlining a possible involvement of the EMT-mediated disruption of the E-cadherin/β-catenin complex in fibrosis. In particular, the immunohistochemical analysis showed the localization of β-catenin in the epithelial cells (where the complex with E-cadherin is located) in the controls and the GED treated mice, while in the DSS mice it was, at least in part, localized in the nuclei. Confocal analyses of E-cadherin and β-catenin confirmed that β-catenin was, at least in part, localized in the nucleus, mainly, of epithelial cells. This is compatible with the disruption of the complex that results in β-catenin translocation to the nucleus as a consequence of the Wnt pathway activation, which has been shown to be related to EMT and fibrosis in various organs [41–51]. In normal conditions, free β-catenin is phosphorylated by GSK-3β and targeted for degradation by a multiprotein complex that includes APC/Axin1. According to our results, GSK-3β is not activated in the fibrotic condition (possibly meaning that its signaling is inhibited), thus β-catenin is free to translocate to the nucleus and to promote its pro-fibrotic signaling.

In addition, GSK-3β is strongly activated in the DSS+GED mice group, where the drug reverted the fibrotic phenotype and restored E-cadherin and β-catenin at normal levels. Other than implying a GSK-3β role as an EMT inhibitor in the intestine, this result implies that GSK-3β activity is directly involved with fibrosis development and in fibrosis reversion. In fact there are other recent evidences reported in the literature [14–15], in which GSK-3β inhibition is related to the reversion of fibrosis in lung and kidney. Nevertheless, until now there were not data (to the best of our knowledge) about the role of GSK-3β in intestinal fibrosis, and our results suggest a strong anti-fibrotic role for the kinase. This is not surprising because it must be underlined that in intestinal fibrosis are active unique molecular signaling networks and well-known pro-fibrotic factors (such as IFN-γ) that show an anti-fibrotic activity in other organs [52–54].

Moreover, the absence of GSK-3β activity in the control group indicates that this kinase does not have a protective role against intestinal fibrosis, but it is activated by GED stimulation and it acts in fibrosis reversion, probably in cooperation with other factors. Being GED a PPAR-γ activator and being the latter a well-known anti-fibrotic factor, this could represent the basis for the GSK-3β anti-fibrotic activity. In particular it may act via stabilization and enhancement of PPAR-γ activity, as seen in various experimental models [52–62] where the β-catenin pathway has been shown to inhibit PPAR-γ signaling. Other than allowing the replenishment of the E-cadherin/β-catenin complex, the free-β-catenin phosphorylation by GSK-3β and its consequent disruption by the proteasome may allow PPAR-γ signaling to revert EMT and fibrosis.

In this context, our data support the involvement of the Wnt/β-catenin pathway in intestinal fibrosis, and support the idea that inhibition of the Wnt pathway is necessary for the reversion of intestinal fibrosis induced by PPAR-γ agonists.

Taken together, our results indicate that the EMT process strongly contributes to the development of intestinal fibrosis in DSS-induced chronic colitis and thus it could represent a valid new target for the development of anti-fibrotic drugs, possibly by acting through the induction of GSK-3β activity.

## Supporting information

S1 Fig Raw Data for E-cadherin western blot(1). Western Blot analysis of total E-cadherin protein levels on the three mice groups (H_2_O, DSS, DSS+ GED).
(TIFF)

S2 Fig Raw Data for E-cadherin western blot (2). Western Blot analysis of total E-cadherin protein levels on the five mice groups (H_2_O, H_2_O +GED, DSS+GED+GW, DSS, DSS+ GED). Image 9, indicated with an arrow, was used for Fig 11.
(TIFF)

S3 Fig Raw Data for β-actin of E-cadherin western blot. **(1)** Western Blot analysis of β-actin as internal control of total E-cadherin on the three mice groups (H_2_O, DSS, DSS+ GED).
(TIFF)

S4 Fig Raw Data for β-Actin of E-cadherin western blot. **(2)** Western Blot analysis of β-actin as internal control of total E-cadherin on the five mice groups (H_2_O, H_2_O +GED, DSS+GED+GW, DSS, DSS+ GED). Image 9, indicated with an arrow, was used for Fig 11.
(TIFF)

S5 Fig Raw Data for Nuclear Snail western blot. Western Blot analysis of Snail nuclear protein levels on the five mice groups (H_2_O, H_2_O +GED, DSS+GED+GW, DSS, DSS+ GED). Image 2, indicated with an arrow, was used for Fig 13.
(TIFF)

S6 Fig Raw Data for Nuclear ZEB1 western blot. Western Blot analysis of ZEB1 nuclear protein levels on the five mice groups (H_2_O, H_2_O +GED, DSS+GED+GW, DSS, DSS+ GED). Image 2, indicated with an arrow, was used for Fig 13.
(TIFF)

S7 Fig Raw data for β-actin of Nuclear Proteins western blot. Western Blot analysis of β-actin as internal control of nuclear proteins on the five mice groups (H_2_O, H_2_O +GED, DSS+GED+GW, DSS, DSS+ GED). Image 2, indicated with an arrow, was used for Fig 13.
(TIFF)

S8 Fig Raw data for total β-catenin and β-actin western blot. Western Blot analysis of total β-catenin protein levels on the three mice groups (H_2_O, DSS, DSS+ GED), with β-actin as internal control. Image 1, indicated with an arrow, was used for Fig 12.
(TIFF)

S9 Fig Raw data for Nuclear β-catenin western blot. Western Blot analysis of nuclear β-catenin protein levels on the five mice groups (H_2_O, H_2_O +GED, DSS+GED+GW, DSS, DSS+ GED). Image 2, indicated with an arrow, was used for Fig 13.
(TIFF)

S10 Fig Raw data for phospho GSK-3β, GSK-3β and vinculin western blot. Western blot analysis of phospho-GSK-3β and GSK-3β protein levels on three of the five mice groups (H_2_O, DSS, DSS+GED), with vinculin as internal loading control. The image was used for Fig 14.
(TIFF)
